# Quantifying Carbon Emissions Generated by Monorail Transits: A Life Cycle Assessment Approach

**DOI:** 10.1155/2022/3872069

**Published:** 2022-03-24

**Authors:** Teng Li, Eryu Zhu

**Affiliations:** Department of Civil Engineering, Beijing Jiaotong University, No. 3 Shangyuancun, Beijing 100044, China

## Abstract

The use of rail transits results in the generation of a large amount of carbon emissions. Throughout the life cycle of a rail transit system, huge amounts of carbon are emitted, which contributes to the threat posed by carbon emission on the city ecosystem. Despite the many methods previously proposed to quantify carbon emissions from rail transit systems, a method that can be applied to measure carbon emissions of monorail systems is yet to be developed. We have used the life cycle assessment (LCA) method to propose a method that can be used to quantify carbon emissions from monorail transits. The life cycle of a monorail transit system was divided into four stages (production, construction, use, and end-of-life). A monorail transit line segment in Chongqing, China, was selected for a case study. The results show that the “use” stage of the monorail transit line system significantly increases (93.2%) carbon emissions, while the “end-of-life” stage does not contribute significantly to the total carbon emitted. The processes of generation of steal, concrete, and cement are the three leading processes that contribute to the emission of carbon dioxide. The percentages of carbon emitted during these processes are 32%, 29.6%, and 13.3%, respectively. Prestressed concrete activity accounts for the largest proportion (91.1%) of the total carbon emissions. The results presented herein can potentially help in realizing sustainable development and developing green transportation.

## 1. Introduction

Global climate changes have aroused great concern worldwide as they have seriously affected social sustainability [1]. One important way to address the problem of climate change is to reduce carbon emissions [2]. The transportation sector facilitates human travel and helps in economic development. However, a large amount of energy is consumed during transportation, resulting in substantial carbon emissions. It has been reported that the transportation sector accounts for 14% of total carbon emissions worldwide [3]. Moreover, carbon emissions from the transportation sector have increased by 29% from 1990 to 2009 [4].

The monorail system uses a single rail instead of two rails as used in traditional rail systems during operation [5]. The monorail systems are low-noise systems that are safe to use. They are characterized by good climbing ability and small turning radii [6, 7]. At present, monorails are in operation in many countries worldwide, such as Japan, Germany, and the United States of America. Egypt, Thailand, Brazil, China, and a few other countries are actively building their monorail systems. This provides a glimpse into the great potential for further advances of monorail transits in the future. Huge quantities of raw materials (such as cement, concrete, and steel) are required for the efficient development of infrastructure required to build the monorail systems. The production of these raw materials is often accompanied by an enormous amount of carbon emissions. As large-scale construction of monorail systems will be realized in the near future, it is necessary to quantify carbon emissions to realize sustainable development.

Life cycle assessment (LCA) is a method of assessing the impacts exerted by products on the environment during their lifetime [8]. In general, process-based LCA consists of four steps: (1) goal and scope definition, (2) inventory analysis, (3) environmental impact assessment, and (4) interpretation [8]. The LCA method has been widely used to evaluate the environmental performance of rail transits in recent years (Table 1).

Table 1 presents the data and research contexts of 25 selected works in which LCA was applied to research into transport systems. Among these 25 selected studies, 12 articles focused on HSR systems, 9 on metro or subways, and 6 on railways. Results obtained by studying light rail transits (LRTs) were reported in two papers. To the best of our knowledge, there are no reports on the carbon emissions from monorail transit systems. It has also been observed that the life cycle has been described and categorized differently by different research groups. Researchers chose the length of the life cycle based on the characteristics of the system. The results obtained in different cases were different. Researchers analyzed databases from their own country or nearby countries to match their local situation. For example, CLCD is generally used as the database for Chinese research. The object of research considered in this paper is a monorail transit in Chongqing, China. Hence, CLCD was selected as the database.

Table 1 demonstrates that LCA can provide a systematic framework to evaluate the life cycle environmental impacts of various rail transit systems. However, there are some research gaps:

1. To date, researchers have widely focused on metro and HSR. To the best of our knowledge, carbon emission has not been quantified from the perspective of the whole life cycle for the case of monorail transit.
2. Researchers have widely studied the four stages of rail transit systems (i.e., production, construction, use, and end-of-life), but a detailed study on the carbon emissions caused by materials production and construction works in the maintenance stage of the rail transit systems has not been conducted.

The aim of the present work is to quantify carbon emissions attributable to monorail transit systems using an LCA approach, with a monorail transit line in Chongqing, China, as a case study. The research work here is organized in four sections.  Section 1 provides a brief introduction to the Chongqing monorail line 2 in China.  Section 2 briefly introduces the methodologies of the LCA calculation. In Section 3, the case study for calculating the carbon emissions during the four stages of a monorail transit line in Chongqing is presented; the calculation results are interpreted; the observations are discussed; the uncertainty analysis and sensitivity analysis are conducted; recommendations are given. In section 4, the conclusions are derived and a summary of the key findings are presented. The results presented are expected to serve as a source of information and data that can be used to conduct LCAs in the future.

## 2. Materials and Methods

This study is based on a process-based LCA method. The different steps involved in the execution of the LCA method are defined in ISO 14040 [8]: goal and scope definition, life cycle inventory analysis, environment impact analysis, and interpretation. The results obtained following the LCA method reveal the potential environmental impacts of the monorail system (from cradle to grave). The methodology is shown in Figure 1.

### 2.1. Goal and Scope: Definition

The goal of this study is to assess the carbon emissions of a monorail transit line segment during the whole life cycle of its operation. The system boundary of the monorail transit was defined based on the guidelines presented in the EN 15978 standard [34]. Specifically, the process is divided into the production (associated with the extraction and upstream production, transport to a factory, and manufacturing processes), construction (associated with the processes of transportation to the working site and installation), use (associated with the use, maintenance, repair, and replacement of the system and the usage of operational energy), and end-of-life (associated with the processes of demolition, material transport, waste processing, and disposal) stages. The basic assumptions made have been presented:

1. The life cycle length of the system is 50 years. The lifespan is the same as the lifespan assumed in previous works on a Chinese subway [22] and a light rail case [33].
2. Vehicles were absent from the system, and this could be attributed to the lack of data. Studies have been previously conducted under similar situations, and the results have been reported [17, 19–22, 26–31].
3. All the wastes are landfilled, and carbon emissions caused by waste transportation during the process of waste processing and waste disposal are primarily considered.
4. Operational energy consumption remains the same every year (this assumption helps simplify the calculations).
5. All the materials are locally available, and the transportation distance is 50 km.

The detailed system boundary is illustrated in Figure 2.

### 2.2. Inventory Analysis

The second step in LCA involves the process of inventory analysis. In this step, information on carbon emission factors associated with different materials and resource (material and energy) consumption at all stages is collected.

#### 2.2.1. Carbon Emission Factors

We chose data presented in the Chinese Core Life Cycle Database (the most authoritative database for LCA in China) [35] to conduct our research to effectively reflect the Chinese conditions. The baseline emission factors of China's regional power grid (from 2011 to 2017) in Chongqing were obtained based on the data from the Ministry of Ecology and Environment of the People's Republic of China [36].

#### 2.2.2. Materials and Energy

Data on material consumption is obtained from construction files, which contain information on the types and quantities of materials used. The Budgetary Norm of Highway Project (JTGT_3832-2018) [37] is studied to determine the machine-teams involved in the different working activities occurring in the construction stage and during the process of demolition associated with the end-of-life stage. The Budget Norm of Maintenance and Strengthening of Highway Bridges (YNG/T B02-2011) [38] is considered to determine the machine-teams involved in the maintenance works associated with the use stage. The data presented in the Expense Standard of Machine-Team of Highway Project (JTGT_3833-2018) [39] are analyzed to obtain the unit energy consumption of different machine-teams. The China Urban Rail Transit Almanac 2019 [40] is referred to, to determine the amount of electricity consumed by the monorail transit lines and stations. The carbon emissions of the monorail transit line are obtained by multiplying the electricity carbon emission factors with the total quantity of electricity.

### 2.3. Environmental Impact Assessment

The third step involves environmental impact assessment or life cycle impact assessment [41]. Results obtained using the various analytical methods reveal that carbon emission (for monorail transits) is realized in four stages. Total carbon emission is calculated using the following equation:

(1) $$\begin{array}{c} C_{tot}=C_{\text{PD}}+C_{\text{CS}}+C_{\text{US}}+C_{\text{EL}}, \end{array}$$

where *C*_*tot*_, *C*_PD_, *C*_CS_, *C*_US_, and *C*_EL_ correspond to the amounts of carbon emitted during the life cycle, the production stage, the construction stage, the use stage, and the end-of-life stage, respectively.

The amount of carbon emissions produced in the production stage is equal to the carbon emission factors of various materials multiplied by the corresponding material quantities. This can be represented by the following equation:

(2) $$\begin{array}{c} C_{\text{PD}}=\sum_{i}{\text{CF}}_{\text{MF},i}\times Q_{\text{MF},i}, \end{array}$$

where CF_MF,*i*_ represents the carbon emission factors of the *i* − *th* material and *Q*_MF,*i*_ represents the consumed quantities of the *i* − *th* material.

Carbon emissions produced during the construction stage are primarily generated during the transportation of the construction materials and consumption of energy (by different construction machines). The amount of carbon emissions generated in the construction stage can be represented by the following equation:

(3) $$\begin{array}{c} C_{\text{MC}}=\sum_{i}{\text{CF}}_{mt,i}\times Q_{mt,i}\times D_{i}+\sum_{i}{\text{CF}}_{cf,i}\times Q_{cf,i}+{\text{CF}}_{e}\times Q_{ce}, \end{array}$$

where CF_*mt*,*i*_ represents the carbon emission factor for the *i* − *th* construction material transportation mode, *Q*_*mt*,*i*_ represents the quantity of the *i* − *th* transported construction materials, and *D*_*i*_ represents the distance between the production factory and the construction site. Here, it is assumed that road freight is the only transportation mode adopted. CF_*cf*,*i*_ represents the carbon emission factor of the *i* − *th* consumed fuel mode in the construction stage, *Q*_*cf*,*i*_ represents the quantity of the *i* − *th* fuel consumed in the construction stage, CF_*e*_ represents the regional carbon emission factor for electricity, and *Q*_*ce*_ represents the quantity of electricity utilized by the construction machines during the construction stage.

The carbon emissions during the use stage are primarily generated during maintenance works and the consumption of electricity by the vehicles and stations. The amounts of the carbon emissions produced during the use stage can be determined using the following equation:

(4) $$\begin{array}{c} C_{\text{US}}=C_{op}+C_{mt}, \end{array}$$

where *C*_US_ represents the amount of carbon emissions generated from the monorail line in the use stage, *C*_*op*_ represents the carbon emissions produced during the operational phase, and *C*_*mtp*_ represents the carbon emissions produced during the maintenance phase.

(5) $$\begin{array}{c} C_{op}=C_{sy}\times \text{Y,} \end{array}$$

(6) $$\begin{array}{c} C_{sy}={\text{CF}}_{e}\times Q_{oe}. \end{array}$$

In (5) and (6), *C*_*sy*_ represents the annual carbon emissions generated from the monorail line in the course of its operation, *Y* is the service life in the operational stage, and *Q*_*oe*_ represents the amount of electricity consumed during the operational stage.

In the maintenance phase, the origin of carbon emissions can be attributed to the processes of material production and fuel consumption (consumed by construction machines). The amount of carbon emissions produced in the maintenance stage can be calculated using the following equation:

(7) $$\begin{array}{c} C_{mt}=\sum_{i}{\text{CF}}_{mt,i}\times Q_{mt,i}+\sum_{i}{\text{CF}}_{mfc,i}\times Q_{mfc,i}+{\text{CF}}_{e}\times Q_{me}, \end{array}$$

where CF_*mt*,*i*_ represents the carbon emission factors of the *i* − *th* material, *Q*_*mt*,*i*_ represents the consumed quantities of the *i* − *th* material, CF_*mfc*,*i*_ represents the carbon emission factor for the *i* − *th* consumed fuel (consumed by machines during the maintenance process), *Q*_*mfc*,*i*_ indicates the quantity of the *i* − *th* fuel consumed (realized during the maintenance process), and *Q*_*me*_ represents the quantity of electricity utilized by the construction machines during the maintenance process.

The carbon emissions generated during the end-of-life stage are produced during the consumption of energy by the construction machines during the processes of demolition and waste transportation. The amount of carbon emission produced during the end-of-life stage can be calculated using the following equation:

(8) $$\begin{array}{c} C_{\text{EL}}=\sum_{i}{\text{CF}}_{f\;d,i}\times Q_{f\;d,i}+{\text{CF}}_{e}\times Q_{de}+\sum_{i}{\text{CF}}_{dm\;t,i}\times Q_{dm\;t,i}\times D_{i}, \end{array}$$

where CF_*f*  *d*,*i*_ represents the carbon emission factor corresponding to the consumed fuel mode (disposal process), *Q*_*fc*,*i*_ represents the quantity of the *i* − *th* fuel consumed during the disposal process, *Q*_*de*_ refers to the quantity of electricity utilized by the construction machines during the disposal process, CF_*dm*  *t*,*i*_ represents the carbon emission factor for the *i* − *th* disposal transportation mode, *Q*_*dm*  *t*,*i*_ represents the quantity of the *i* − *th* transported materials, and *D*_*i*_ indicates the distance between the construction site and the disposal area.

### 2.4. Interpretation

In this step, the conclusions are arrived at based on the results obtained during inventory analysis and impact assessment. The key stages, working activities, and materials (used throughout the life cycle) that affect the extent of carbon emission produced during the functioning of a monorail transit were identified. The uncertainty analysis and sensitivity analysis methods were used, and the data were analyzed using Oracle Crystal Ball software to determine the possible range of life cycle carbon emissions of a monorail transit. The parameters that affect the results are also identified.

## 3. Results and Discussion

### 3.1. Monorail Transit Line: Background Information

The monorail transit line 2 in Chongqing, China, is selected for a case study to demonstrate and validate the proposed LCA approach. It was inaugurated in December 2004 as the first straddle monorail line in China. It is one of the two straddle monorail lines that are currently in operation in China. Its operational mileage has reached 31.36 km. We have selected a section (from Niujiaotuo to Daping; length: 2409.09 m) of the entire route for our studies. We have quantified the carbon emissions produced in the selected section. The specific route under consideration is shown in Figure 3.

### 3.2. Calculating Carbon Emissions: Results

#### 3.2.1. Carbon Emissions in the Production Stage

According to equation (2), the carbon emissions produced during the production of the materials primarily used for production are shown in Table 2.

The total amount of carbon emissions produced during the production of main materials was 3,365.43 t.

#### 3.2.2. Carbon Emissions Produced during the Construction Stage

The carbon emissions produced during the construction stage are primarily generated during the processes of material transportation and construction. Equation (3) and the assumptions made were taken into consideration to calculate the amount of carbon emissions produced during the process of transportation of the materials (Table 3).

The total amount of carbon emissions produced during the transportation of materials was 113.49t. The amount of carbon emissions produced during the process of on-site construction was calculated (equation (3), Table 4). The carbon emission factors corresponding to electricity and diesel are 1.294 t CO_2_/MWh and 3.664 kg/kg, respectively.

The amount of carbon emissions produced in the area of the chosen line segment was calculated to be 5,653.58 t. When the amount of carbon emissions produced during the transportation of the main material is taken into account, the total amount of carbon emissions generated during the construction stage is calculated to be 5,767.18 t.

#### 3.2.3. Carbon Emissions Produced during the Maintenance Phase of the Use Stage

The assumptions were taken into account, and the carbon emissions produced during the maintenance phase were calculated (equation (7), Table 5). The guidelines presented in the Budget Norm of Maintenance and Strengthening of Highway Bridges (YNG/T B02-2011) [38] were followed, and it was assumed that each time, one concrete treatment, 100 m-long expansion joint, 10 dm^3^-volume bearings, 1000 m-long cracked concrete, and 400 m^3^-area concrete beam section were maintained. According to the Budget Norm of Maintenance and Strengthening of Highway Bridges (YNG/T B02-2011) [38], the maintenance works are carried out once every ten years.

The total amount of carbon emissions produced during material, electricity, and fuel consumption during the construction of the machine was calculated to be 16.87 t/10 years. If the life cycle is considered to be 50 years long, the total carbon emission is calculated to be 60.51 t.

#### 3.2.4. Amount of Carbon Emissions Produced during the Operation Phase of the Use Stage

The data presented in the Ministry of Ecology and Environment of the People's Republic of China [36] was analyzed to determine the baseline emission factors corresponding to the regional power grid in China. The data for different years were collected, and the carbon emission factors of different regions (time range: 2006–2017) were determined. Chongqing is situated in central China. The ARMA time series method was used to predict the electricity carbon emission factors of central China (for the years spanning 2002–2018) based on the existing data, as data for the years before 2006 and after 2017 were unattainable. The forecast results for 2002 and 2018 are 1.294 t CO_2_/MWh and 0.5907 t CO_2_/MWh, respectively.

The annual power consumption amounts and the annual passenger turnover were determined by analyzing the statistical data presented in the China Urban Rail Transit Yearbook 2019 [40]. The amount of carbon emission produced was calculated accordingly. The amount of carbon emissions produced by monorail line 2 (during its operation in 2018) was calculated to be 34,029.22 t. The total amount of carbon emissions produced during the 50-year-long life cycle was calculated to be 1,701,461 t. The amount of carbon emissions produced per unit length was 54255.77 t/km. The amount of carbon emissions produced by the chosen part of line 2 (length: 2.4 km) was 130,213.85 t. Equation (4) was used to calculate the total amount of carbon emissions generated during the whole use stage. The amount was calculated to be 130,274.36 t.

#### 3.2.5. Carbon Emissions Produced during the End-of-Life Stage

Equation (8) was used, and the assumptions made were considered to calculate the amount of the carbon emissions produced during the process of structure demolition and waste disposal during the end-of-life stage. The engine-driven air compressor within 9 m^3^/min was primarily used during the demolition process. The total amount of energy consumed during the demolition process was calculated to be 11,916.83 kWh. The total amount of carbon emissions generated during the demolition process was calculated to be 356.35 t. The total amount of carbon emissions generated during the process of waste transportation was calculated to be 113.49 t, and the total amount of carbon emissions produced during this stage was 469.84 t.

### 3.3. Amount of Carbon Emissions Produced during Different Stages

A comparison of the amounts of carbon emissions produced during different stages of the life cycle of the material is presented in Figure 4(a) and Figure 4(b). Analysis of the figures indicates that the maximum amount of the carbon emissions generated during the life cycle of the monorail transit is produced during the use stage (93.2%). The amount produced in this stage is significantly higher than the amount produced during the other stages. This can be primarily attributed to the fact that the amount of carbon emissions produced during the process of energy consumption during the entire 50-year-long operation period is considered during the study of the operational phase. A huge amount of carbon emissions is produced during this phase. Various maintenance works are carried out during the life cycle of the material. Each stage requires a certain amount of manpower and materials for completion. Different types of machinery are also required for the effective execution of the process. Maintenance work is carried out once every 10 years. Thus, a total of five maintenance cycles are carried out during the whole life cycle. This results in the generation of a large amount of carbon emissions in the use stage. A considerable amount of carbon emissions is also produced during the construction stage (4.1%). This can be attributed to the fact that a huge quantity of energy is consumed by different working machines during this process. The amount of carbon emissions generated during the production stage (2.4%) is slightly lower than the amount generated during the construction stage. It has also been observed that the amount of carbon emissions generated from the end-of-life stage is only 0.3% of the total amount generated, an insignificant amount as compared to emissions produced in other stages.

### 3.4. Carbon Emissions from Different Materials

Figures 5(a) and 5(b) provide a comparison of the amounts of carbon emissions produced during the use of different materials. As the figures show, there are significant differences in the amount of carbon emissions generated by different types of materials. The top 11 construction materials that contribute the most toward the production of carbon emissions are listed in Figure 5(a). The cumulative amount of the carbon emissions generated by these 11 materials is 3365.15 t, accounting for almost all of the total carbon emissions generated during the production stage. Specifically, the use of steel (32%), concrete (29.6%), cement (13.3%), and mortar (13%) results in the production of the maximum amount of carbon emissions during the production stage.

This can be attributed to the fact that a monorail line is a reinforced concrete structure that requires the use of a large amount of steel (1,376.36 t), concrete (3,549.61 m^3^), cement (622.3 t), and mortar (1,144.91 m^3^). The corresponding carbon emission factors are significantly high. The total amount of carbon emissions produced is large as the consumption and carbon emission factors of these materials are significantly high. Therefore, the key to improving the environmental performance of monorail transit lies in decreasing the amount of carbon emissions generated by these materials. It has been previously reported [42] that an efficient water reducing agent can be used to replace cement during the process of concrete production. This can help in reducing the amount of carbon emissions produced during the material production stage. The concrete strength can be improved simultaneously to reduce the amount of cement and concrete used. Furthermore, designers could consider using more amounts of renewable construction materials (such as renewable concrete) in the design stage [43]. Mortar, bricks, building blocks, gravel, sand, and other materials also contribute to the generation of carbon emissions in the production stage. The use of these materials results in the generation of insignificant amounts of carbon emissions.

### 3.5. Carbon Emissions: Analysis of Working Activities Occurring in the Construction Stage

A comparison of the amounts of carbon emissions generated at different stages of the construction stage is presented in Figure 6. Fifteen working activities are considered. The results reveal that prestressed concrete activity accounts for the largest proportion (91.1%) of the total carbon emissions produced in this stage. The amount of carbon emission produced during prestressed concrete activity is significantly higher than the amount produced during other construction activities. This can be primarily attributed to the fact that a huge quantity of electricity is consumed during the operation of machines single-cylinder slow-motion winch within 30 KN (2,681,021.27 kWh), single-cylinder slow-motion winch within 50 KN (934,667.96 kWh), Φ100 mm electric multistage water pump (≤120 m; 204,479.87 kWh), and concrete delivery pump (60 m^3^/h; 98,556.12 kWh). In addition, a considerable amount of carbon emissions is generated during the construction of the beam concrete (3.6%). The amount of carbon emissions generated during the processes of beam reinforcement (1.5%) and rebar processing (1.5%) is slightly lower than the amount produced during the process of beam concrete construction. The amount of carbon emissions attributable to other construction activities accounts for less than 1% of the total carbon emissions originating from all construction activities. This indicates that these activities do not significantly affect the environment.

### 3.6. Uncertainty Analysis: Construction Stage and Production Stage

The uncertainty of carbon emissions corresponding to material and fuel consumption can be attributed to construction errors. Uncertainty analysis was conducted using the Oracle Crystal Ball (Figure 7) to evaluate the possible range of carbon emissions for a monorail segment during its life cycle. Standard normal distributions were assumed for the input parameters, and the number of testing times was set to 100,000. The probability distributions corresponding to the target variables were normal distributions. The variation range calculated for carbon emissions was 100,000–180,000 t.

### 3.7. Life Cycle: Sensitivity Analysis

The Oracle Crystal Ball was used to determine the sensitivity of carbon emissions during the life cycle of the monorail transit line. The results are shown in Table 6.

Analysis of the data presented in Table 6 reveals that the length of the life cycle, amount of electricity consumed annually, single-cylinder slow-motion winch within 30 KN quantity, single-cylinder slow-motion winch within 50 KN quantity, use of C40 concrete quantity, cement mortar (1 : 3) quantity, and brick 200 × 95 × 53 quantity are the sensitive factors that affect the final carbon emission results. The length of the life cycle and the amount of electricity consumed annually during the operation of the system significantly influence the amount of carbon emission produced by the monorail system during its lifetime. In addition, the quantities of single-cylinder slow-motion winch within 30 KN, single-cylinder slow-motion winch within 50 KN, C40 concrete, cement mortar (1 : 3), and brick 200 × 95 × 53 also exert a certain influence on the results. It was observed that the degrees of influence were almost the same.

### 3.8. Discussion of the Approach

This calculation framework can be used to calculate the amount of carbon emission produced by a monorail line during its lifetime, but it can also be used to calculate the amount of carbon emissions produced by ordinary railway, light rail, subway, and other rail transportation systems. The calculation results can help design the monorail transit system, and the results can help reduce the amount of carbon emission produced at the initial stages of the process.

As there are few monorail lines in operation in China, it is difficult to obtain field data. It is challenging to verify the universality of the results calculated from the only data available. More data can be obtained in the future as the construction of monorail traffic has been planned. Our model will be further optimized to make it universal.

### 3.9. Recommendations for Future Research

More attention should be paid to the following research directions:

1. Verification and application of the approach used by us should be realized by analyzing fundamental data. Therefore, attention should be paid to obtaining more amounts of data to improve the developed approach.
2. Some scenarios can be designed to simulate the carbon emission reduction effects based on the calculation results presented. This can potentially help in proposing helpful suggestions that can be exploited by designers and politicians for the sustainable development of the city.

## 4. Conclusions

We calculated the amount of carbon emissions produced during the operation of a monorail transit line (during its lifetime) using the LCA method. A segment of the Chongqing monorail line 2 was selected for the case study for validating the developed model. The following conclusions were drawn:

1. The life cycle of the monorail transit line can be theoretically divided into four stages: the production, construction, use, and end-of-life stages. The use stage contributes >90% of the carbon emissions produced during the lifetime of the monorail transit line. A significant amount of carbon emissions is produced during the construction and production stages. The amount of emissions produced during the end-of-life stage is less than the amount produced in the other three stages.
2. Steel, concrete, and cement are the most important sources of carbon emissions.
3. Prestressed concrete activity accounts for the maximum proportion (91.1%) of the total carbon emissions. Significant amounts of carbon emissions are generated during the process of beam concrete construction (3.6%). The amounts of carbon emissions generated during the process of beam reinforcement (1.5%) and rebar processing (1.5%) are slightly lower than the amounts generated during the process of beam concrete construction.

In summary, the results presented herein can help gain a better understanding of the effects of the monorail transit industry on the ecosystem. The results can potentially help develop ideas that can be used by designers working in the rail transit industry to meet low carbon emission goals.

## Figures and Tables

**Figure 1:** Methodology followed for carbon emission analysis.

**Figure 2:** System boundary.

**Figure 3:** Case scenario.

**Figure 4:** (a) Amounts of carbon emissions generated during different stages of operation throughout the life of the material. (b) Proportion of carbon emissions generated during different life cycle stages.

**Figure 5:** (a) Amounts of carbon emissions generated during the use of different materials. (b) Proportions of carbon emissions generated during the use of different materials.

**Figure 6:** Proportions of carbon emissions generated during different construction activities.

**Figure 7:** Uncertainty analysis conducted for carbon emissions produced during the life cycle of the material.

**Table 1:** LCA and its application in the field of transport.

Reference	Country, region	Type of rail	Lifespan (years)	Function unit	Data	Life cycle stages
[9]	USA	Railway, RTS, subway, and HSR	Varying	PMT and VMT	Sectors and literature	Vehicle (manufacture, operation, maintenance, insurance); infrastructure (construction, operation, maintenance); fuel consumption
[10]	USA	Railway, metro, CR, and LRT	—	PKT	Literature	Train manufacturing, train maintenance, station construction, track construction, station operation, station maintenance, electricity generation supply chains
[11]	USA, California	HSR	—	PKT	SimaPro	Vehicle, station, energy production
[12]	USA, California	HSR	20	PKT	Literature	Vehicle, infrastructure, energy production
[13]	Turkey	HSR and railway	40	PKM	SimaPro 7.3.3	Infrastructure (production of electrical energy, construction of lines, maintenance of lines, operation of lines, waste disposal); operation (production of electrical energy, production of train vehicles, maintenance of train vehicles, operation of train vehicles, waste disposal)
[14]	Italy, Rome	Metro	30	VKT	Operators and GaBi	Material acquisition, manufacturing, use, and end-of-life
[15]	China	HSR	20	SKM	Chinese Core Life Cycle Database (CLCD) and ecoinvent	Vehicle operation, vehicle manufacturing/maintenance/disposal, infrastructure construction
[16]	USA, New Jersey	Commuter	—	1 mile	Literature	Material manufacturing
[17]	Brazil, Rio de Janeiro	Metro	60		IPCC 2006	Infrastructure construction, train manufacture, maintenance, infrastructure operation, and train operation
[18]	Portugal	HSR	35	PKT	SimaPro and ecoinvent	Material, manufacturing, use, disposal
[19]	Austria, Vienna	Subway	100	PKT	Biding documents and GEMIS 4.5	Infrastructure construction, infrastructure operation
[20]	Spain, Bueno	HSR	60	PKM/year, TKM/year	Literature	Infrastructure construction, infrastructure maintenance, operation, 60 years
[21]	Canada, Toronto	Subway	8 (construction time)	Year	Literature, construction data	Infrastructure construction, operation
[22]	China, Shanghai	Metro	50	1 km	Observed data	Materials production, materials transportation, on-site construction, operation, and maintenance, 50 years, 1 km, PKT, VKT
[23]	India, Mumbai	Railway	25	PKT, VKT	Department data	Manufacturing, maintenance and operation, infrastructure construction, infrastructure maintenance
[24]	State of Qatar, Doha	Metro	—	1000 PKT	Company data and GaBi 6.0	Train operations, train stations operation
[25]	Turkey	Railway	—	TKM	SimaPro and ecoinvent	
[26]	China, Shanghai	HSR	100	-	Literature	Conception stage, construction stage, operation and maintenance stage, and disposal stage
[27]	China	HSR	100	T/km T/vehicle	IO-LCA hybrid	Material production, construction
[28]	France	HSR	120	Travel of up to 17 metric tons per axle	Experts and ecoinvent 3.1	Production, maintenance, end-of-life
[29]	Belgium	Railway	6	TKM	Country-specific data and ecoinvent	Transport operation, rail equipment, and infrastructure
[30]	China, Fuzhou	Subway	Construction time	Km	In-service lines, regional database (IKE)	Infrastructure construction
[31]	Spain	HSR	100	Year	Google Earth	Construction, maintenance, one-year operation
[32]	USA, Houston	HSR	60	PKT	Ecoinvent	Raw material extraction and processing, vehicle manufacturing, material distribution, construction, operation and maintenance, and end-of-life
				VKT		
[33]	Turkey, Kayseri	LRT	50	PKM	Company, SimaPro, and ecoinvent	Extraction and production of raw materials, transportation of the raw materials to construction sites, vehicle manufacture, transportation of vehicles, construction of infrastructure, operation, maintenance, and waste disposal

**Table 2:** Carbon emissions generated during the production of materials primarily used for production.

Material	Unit	Quantity	Factor (kg/unit)	Carbon emissions (t)
Cement	t	622.30	719.62	447.82
C20 concrete	m^3^	868.71	201.38	174.94
C25 concrete	m^3^	105.07	250.54	26.32
C30 concrete	m^3^	2,556.20	306.78	784.19
C40 concrete	m^3^	6.04	391.03	2.36
C50 concrete	m^3^	13.59	510.94	6.94
Sand	t	2,195.88	9.57	21.01
Gravel	t	1,728.33	12.69	21.93
Stone	m^3^	35.94	6.05	0.22
Brick 200 × 95 × 53	1000	474.83	504.00	239.31
Building blocks	m^3^	789.65	146.00	115.29
Waterproofing	m^2^	3,088.14	2.37	7.32
Coating	t	41.46	25.00	1.03
Steel Q235B	t	163.85	1,789.06	293.14
Other steel	t	29.97	1,789.06	53.61
Steel plate	t	0.29	1,789.06	0.52
Steel reinforcement	t	408.39	1,789.06	730.63
Wood	m^3^	35.87	10.45	0.37
Aluminum	t	0.78	18.57	0.01
Mixed mortar (M5)	m^3^	236.82	228.03	54.00
Mixed mortar (M2.5)	m^3^	50.10	199.23	9.98
Cement mortar (1 : 1)	m^3^	34.29	730.2	25.04
Cement mortar (1 : 2)	m^3^	43.74	531.52	23.25
Cement mortar (1 : 2.5)	m^3^	252.34	469.41	118.45
Cement mortar (1 : 3)	m^3^	527.62	393.65	207.70
Total				3,365.43

**Table 3:** Carbon emissions produced during transportation of the materials during the construction stage.

Item	Means and energy	Distance (km)	Quantity	Carbon emissions (t)
Steel	Truck, diesel	50	1,376.36 t	4.88
Concrete	Mixer, diesel	50	3549.61 m^3^	68.87
Aluminum	Truck, diesel	50	0.78 t	0.01
Sand and gravel	Truck, diesel	50	3,924.21 t	13.91
Stone	Truck, diesel	50	35.94 m^3^	0.55
Brick	Truck, diesel	50	478.15 m^3^	7.32
Building blocks	Truck, diesel	50	789.65 m^3^	12.08
Wood	Truck, diesel	50	35.87 m^3^	0.55
Coating	Truck, diesel	50	41.46 t	0.16
Cement	Truck, diesel	50	622.3 t	2.41
Mortar	Truck, diesel	50	1,144.91 m^3^	2.75
Total				113.49

The total amount of carbon emissions produced during the transportation of materials was 113.49 t.

**Table 4:** Carbon emissions produced during on-site construction.

Working activities	Item	Construction machine	Energy	Energy consumption	Carbon emissions (t)
Foundation	Earth excavation	Crawler type mechanical single bucket excavator within 1.0 m³	Diesel	1,209.33 kg	4.44
	Stone excavation	Crawler type mechanical single bucket excavator within 1.0 m³	Diesel	766.86 kg	2.81
		Motorized air compressor within 9 m^3^/min	Electricity	1,433.42 kWh	1.66
	Impact drilling pile	Crawler type mechanical single bucket excavator within 1.0 m³	Diesel	114.23 kg	0.42
		Trucks within 10 t	Diesel	310.87 kg	1.14
		Truck crane within 16 t	Diesel	278.41 kg	1.02
		JK8 percussion drill	Electricity	10,157.69 kWh	13.10
		Mud separator	Electricity	74.55 kWh	0.10
		Mud mixer	Electricity	434.89 kWh	0.56
		Mud pump within Φ 100 mm	Electricity	1,275.30 kWh	1.65
		AC arc welder within 42 kV A	Electricity	331.52 kWh	0.43
	Manual digging pile	Single barrel slow winch within 50 kN	Electricity	15,087.19 kWh	19.46

Bridge substructure	Concrete	Concrete delivery pump within 60 m^3^/h	Electricity	18,372.52 kWh	23.70
		Truck crane within 25 t	Diesel	2,868.75 kg	10.53
	Steel	Truck crane within 25 t	Diesel	2,562.28 kg	9.40
		Automatic steel seam welder	Electricity	4,148.22 kWh	5.35
		AC arc welder within 32 kV A	Electricity	9,809.58 kWh	12.65
	Bearing	Truck crane within 20 t	Diesel	206.96 kg	0.21
		AC arc welder within 32 kV A	Electricity	178.36 kWh	0.23

Bridge superstructure	Concrete	Concrete delivery pump within 60 m^3^/h	Electricity	43,544.45 kWh	56.17
		Truck crane within 25 t	Diesel	40,285.13 kg	147.85
	Cast-in-place T-beam reinforcement	AC arc welder within 32 kV A	Electricity	44,693.70 kWh	57.66
		AC butt welder within 150 kV A	Electricity	20,485.11 kWh	26.43
	Centralized and standardized processing of rebar	CNC vertical rebar bending center	Electricity	711.17 kWh	0.92
		AC arc welder within 32 kV A	Electricity	44,693.70 kWh	57.66
		AC butt welder within 150 kV A	Electricity	20,485.11 kWh	26.43
	Prestressed concrete	Concrete delivery pump within 60 m^3^/h	Electricity	98,556.12 kWh	127.14
		Single-cylinder slow-motion winch within 30 kN	Electricity	2,681,021.27 kWh	3,458.52
		Single-cylinder slow-motion winch within 50 kN	Electricity	934,667.96 kWh	1,205.72
		Φ100 mm electric multistage water pump (≤120 m)	Electricity	204,479.87 kWh	263.78
		AC arc welder within 32 kV A	Electricity	51,668.13 kWh	66.65
	Steel strand	Prestressed steel tensile machine	Electricity	2,284.49 kWh	2.95
		Bellows rolling machine	Electricity	571.23 kWh	0.74
	Prestressed reinforcement	Prestressed stretching machine within 900 kN	Electricity	6980.95 kWh	9.01
		Bellows rolling machine	Electricity	621.10 kWh	0.80
		Single-cylinder slow-motion winch within 50 kN	Electricity	6,607.41 kWh	6.61

Other installation	Optical cable laying	Trucks within 10 t	Diesel	134.38 kg	0.49
		Engine-driven air compressor within 17 m^3^/min	Electricity	46.36 kWh	0.06
	Electric cable laying	Trucks within 10 t	Diesel	33.58 kg	0.12
		Truck crane within 5 t	Diesel	9.95 kg	0.04

**Table 5:** Amount of carbon emissions produced during maintenance works.

Working activities	Items	Unit	Quantity	Carbon emission factors	Carbon emissions (t)
Concrete treatment	Polymer mortar	m^3^	2.80	354.75 kg carbon emissions/m^3^	0.99
	Concrete protective coating	kg	33.60	25 kg carbon emissions/t	0.00
	Electric concrete grinding machine within 3 kw	Machine-team	9	5 kWh/machine-team	0.06
	Handheld electric percussion drilling within 3 kw	Machine-team	18	98.28 kWh/machine-team	2.29
	Electric single-stage centrifugal clean water pump within 50 mm	Machine-team	56	23 kWh/machine-team	1.67
	Engine-driven air compressor within 0.3 m^3^/min	Machine-team	15.20	16.1 kWh/machine-team	0.32
	Total carbon emissions	t	5.33		

Expansion joint repair and replacement (per 10 m)	Plain round bar	t	0.01	1789.06 kg/t	0.02
	Steel plate	t	0.05	1789.06 kg/t	0.09
	Petroleum asphalt	t	0.01	174.244 kg/t	0.00
	AC arc welder within 32 kV A	Machine-team	1.90	96.53 kWh/machine-team	0.24
	Total carbon emissions	t	0.35		

Bearing replacement (per 10 dm^3^)	HRB400 steel rebar	t	0.10	1789.06 kg/t	0.18
	Steel plate	t	0.01	1789.06 kg/t	0.02
	AC arc welder within 32 kV A	Machine-team	0.02	96.53 kWh/machine-team	0.00
	Total carbon emissions	t	0.20		

Crack treatment (per 100 m)	Engine-driven air compressor within 0.3 m^3^/min	Machine-team	3.6	16.1 kWh/machine-team	0.08
	Total carbon emissions	t	0.08		

Section enlargement (per 10 m^3^)	C30 pump concrete	m^3^	15	306.78 kg/m^3^	4.60
	32.5 cement	t	7.65	719.62 kg/t	5.51
	Medium (coarse) sand	m^3^	8.85	9.57 kg/m^3^	0.08
	Gravel	m^3^	8.40	12.69 kg/m^3^	0.11
	Concrete mixer within 250 L	Machine-team	1.24	20.91 kWh/machine-team	0.03
	4–6 m^3^/h concrete jet	Machine-team	3.17	15.4 kWh/machine-team	0.06
	Engine-driven air compressor within 9 m^3^/min	Machine-team	2.78	51.50 kg diesel/machine-team	0.52
	Total carbon emissions	t	10.91		

**Table 6:** Sensitivity analysis conducted for carbon emissions produced during the production stage.

Order	Parameters	Variance contribution (%)	Rank correlation
1	Life cycle length	47.0	0.69
2	Annual operation electricity consumption	46.9	0.68
2	Single-cylinder slow-motion winch within 30 KN	0.1	0.02
3	Single-cylinder slow-motion winch within 50 KN	0.1	0.01
4	C40 concrete quantity	0.1	0.01
5	Cement mortar (1 : 3) quantity	0.1	0.01
6	Brick 200 × 95 × 53 quantity	0.1	0.01
7	Others	0.1	-

## Data Availability

The data used to support the findings of this study are available from the corresponding authors upon request.

## Abbreviations

ARMA: Autoregressive moving average
CE: Carbon emissions
CEF: Carbon emission factor
GHG: Greenhouse gas
HSR: High-speed rail
IO: Input-output
LCA: Life cycle assessment
LRT: Light rail transit
PKT: Passenger kilometer traveled
VKT: Vehicle kilometer traveled
PMT: Passenger mile traveled
RTS: Rapid transit system
SKM: Per seat per kilometer traveled
VMT: Vehicle mile traveled.
